The article "Glaucoma Detection Using Image Processing and Supervised Learning for Classification" was published in 2022. Journal: J Healthc Eng.

# Glaucoma Detection Using Image Processing and Supervised Learning for Classification

**DOI:** 10.1155/2022/2988262

**Published:** 2022-03-01

**Authors:** Shubham Joshi, B. Partibane, Wesam Atef Hatamleh, Hussam Tarazi, Chandra Shekhar Yadav, Daniel Krah

**Affiliations:** ^1^Department of Computer Engineering, SVKM'S NMIMS MPSTME Shirpur, Shirpur 425405, Maharashtra, India; ^2^Department of ECE, SSN College of Engineering, Chennai, India; ^3^Department of Computer Science, College of Computer and Information Sciences, King Saud University, P.O. Box 51178, Riyadh 11543, Saudi Arabia; ^4^Department of Computer Science and Informatics, School of Engineering & Computer Science, Oakland University, Rochester Hills,MI,USA 318 Meadow Brook Rd, Rochester, MI 48309, USA; ^5^Ministry of Electronics and Information Technology, Delhi, India; ^6^Tamale Technical University, Tamale, Ghana

## Abstract

A difficult challenge in the realm of biomedical engineering is the detection of physiological changes occurring inside the human body, which is a difficult undertaking. At the moment, these irregularities are graded manually, which is very difficult, time-consuming, and tiresome due to the many complexities associated with the methods involved in their identification. In order to identify illnesses at an early stage, the use of computer-assisted diagnostics has acquired increased attention as a result of the requirement of a disease detection system. The major goal of this proposed work is to build a computer-aided design (CAD) system to help in the early identification of glaucoma as well as the screening and treatment of the disease. The fundus camera is the most affordable image analysis modality available, and it meets the financial needs of the general public. The extraction of structural characteristics from the segmented optic disc and the segmented optic cup may be used to characterize glaucoma and determine its severity. For this study, the primary goal is to estimate the potential of the image analysis model for the early identification and diagnosis of glaucoma, as well as for the evaluation of ocular disorders. The suggested CAD system would aid the ophthalmologist in the diagnosis of ocular illnesses by providing a second opinion as a judgment made by human specialists in a controlled environment. An ensemble-based deep learning model for the identification and diagnosis of glaucoma is in its early stages now. This method's initial module is an ensemble-based deep learning model for glaucoma diagnosis, which is the first of its kind ever developed. It was decided to use three pretrained convolutional neural networks for the categorization of glaucoma. These networks included the residual network (ResNet), the visual geometry group network (VGGNet), and the GoogLeNet. It was necessary to use five different data sets in order to determine how well the proposed algorithm performed. These data sets included the DRISHTI-GS, the Optic Nerve Segmentation Database (DRIONS-DB), and the High-Resolution Fundus (HRF). Accuracy of 91.11% for the PSGIMSR data set and the sensitivity of 85.55% and specificity of 95.20% for the suggested ensemble architecture on the PSGIMSR data set were achieved. Similarly, accuracy rates of 95.63%, 98.67%, 95.64%, and 88.96% were achieved using the DRIONS-DB, HRF, DRISHTI-GS, and combined data sets, respectively.

## 1. Introduction

Imaging, analysis, and computer vision approaches are becoming more popular across all fields of medical research, but they are especially essential in the field of ophthalmology today. Ophthalmology is, without a doubt, a multifaceted field, both in terms of research and therapeutic application. In recent years, medical imaging has grown to become prominent owing to the rapid advancements achieved in computerized medical image reconstruction, as well as the accompanying developments in analytic techniques and computer-aided diagnosis (CAD). The use of medical images has become more significant in the identification and diagnosis of a broad variety of diseases and medical conditions. Imaging techniques for medical imaging are being researched with the detachment of the production of computer utensils that will assist in the measurement and visualization of illness and functional constructions in the body. Medical digital imaging has developed as a vital component of today's health-care procedures, and it will continue to grow in importance.

One of its most valuable features is the capacity to retrieve data on a wide range of diseases from patients' visual documentation and permanent medical history. An imaging system of the highest quality is vital for future medical decision-making and reducing unnecessary medical procedures. As digital photography and processing power have improved, so has ophthalmology as a field. As digital imaging and processing capabilities improve, so do the possibilities for employing digital imaging and processing in the field of ophthalmology. Because of this, image processing is increasingly being seen as a key component of scientific research and development in the sciences and technology. Many computer-aided design techniques have been developed to aid in the interpretation of medical pictures so that more trustworthy and accurate diagnoses may be made. By adopting computer-aided design (CAD), medical imaging technicians might be assisted in their analysis by specialist computer systems. Recent studies demonstrate that the CAD system can improve diagnostic accuracy while simultaneously decreasing tiredness, lowering the number of missed diseases due to exhaustion or ignored data, and enhancing the variability between readers. CAD systems have the potential to provide an alternative to mass screening programmes that must analyze a large number of fundus pictures as quickly as feasible.

The use of fluorescent dye angiography (FA) and optical coherence tomography (OCT) in conjunction with clinical examination and fundus photography may aid in the analysis of glaucoma [1], in addition to the traditional methods of examination and fundus photography. Angiograms using fluorescein dye are a type of diagnostic procedure in which an intravenous injection of a fluorescent dye is administered to a patient's systemic circulation, and the fluorescent properties of the dye are activated by shining a specific wavelength of light into the patient's eye while the dye is being administered. A 2D cross-sectional image of ocular tissue structures is produced using optical coherence tomography (OCT), with dimensions specified by the spread way of bright and a vertical three-dimensional way. Due to the fact that OCT images are made up of several axial scans, it is feasible to produce a computational three-dimensional reconstruction of the retina by stitching together several OCT images. A fundus camera is used in the performance of fluorescein angiography, which is referred to as fluorescein angiography when performed by an ophthalmologist.

When utilized as a primary population screening tool, new imaging technologies in retinal image processing need employment and are thus prohibitively expensive when used. It is thus necessary to create a less luxurious method for the detection of eye illnesses, the monitoring of disease progression, and the implementation of a mass screening programmed to identify people who are at risk of acquiring eye diseases. Early detection of the condition by regular screening and prompt action would be critical in effectively managing the course of the illness. In this study, the goal is to diagnose glaucoma in monocular fundus photographs by using feature extraction techniques to them.

Progressive optic neuropathy (POAG) is a progressive optic neuropathy that occurs as a consequence of tissue loss in the neuroretina edge of the ocular CD (OD), with a resultant upsurge in the size of the ocular cup as a result of this tissue loss. It is common practice to consider the CDR throughout the assessment process when examining fundus photographs for glaucoma. The CDR is one of the most important physiological features for diagnosing and treating eye illness and is therefore taken into consideration throughout the assessment process. When two optic nerves have the same CDR but differing neuroretina rim width, the asymmetries of cup-to-disc may be induced by a variety of illnesses and are more susceptible to restrictions with interindividual variability than when two optic nerves have the same CDR but unequal neuroretina rim width. A further point to mention is that the optical density (OD) size is not a reliable diagnostic tool for glaucoma. Blood vascular interruption is one of the most difficult parts of segmenting the optic cup and disc with greater dependability and precision, and it represents one of the most difficult challenges. Glaucoma progresses in a way that causes the optic cup to get larger, resulting in differences between the fundus images of the afflicted and unaffected eyes. It is thus necessary to perform an efficient and exact segmentation of the OD and optic cup in order to assess the pattern of rim loss, estimate quantitative parameters, and detect the morphological indications of glaucoma in the eyeball, among other things. Physiological changes in the eye must be shown in fundus photographs in order to identify changes in the eye's structural and functional abnormalities over time. This is necessary in order to illustrate the variability and progression of glaucoma over time.

The goal of this study is to improve classification accuracy by automatically classifying photos of normal and glaucoma eyes based on fundus images' histograms, textures, and fractals. For increased accuracy, it is required to study and choose critical criteria for glaucomatous image categorization that are more specific and sensitive than the standard now in use. With computer-aided methods for retinal image analysis, the reproducibility and objectivity of eye-quality evaluations can be improved. There must be an accurate description of the optic nerves' optical impression to accurately diagnose and set a baseline from which changes may be discovered by examination, according to the ophthalmologist. Detecting changes in the disease's progress and avoiding future vision loss are the goals of this study on glaucoma, a potentially blinding condition. In the early days of glaucoma diagnosis, a quantitative categorization of the optic nerve using the CDR was the most widely used, and it remains so today. CDR, despite its many advantages, such as its simplicity of use and the absence of magnification aberrations, has two fundamental limitations that restrict its accuracy. Glaucoma-induced damage to the optic disc (OD) has been shown to be characterized by the CDR in an inconsistent manner. The CDR does not take the disc's diameter into consideration, which leads to a high number of FP and FN prints. In glaucoma, the most basic change is the loss of neuroretina rim tissue, rather than CDR.

Disc size is not taken into account in the CDR staging approach, and focal constriction of the neuroretina rim is not adequately stressed in the system, which are the two most major weaknesses of the procedure. Taking these elements together, the CDR's utility in terms of diagnostic accuracy is diminished. Another item to consider is that CDR does not readily detect the localized changes in the neuroretina rim that are so indicative of glaucoma. This is the second point to examine.  Figure 1 displays two optic nerves with cups and discs that are comparable in size, but the CDR is the same in each of the examples. Although the vertical CDR on both wheels is the same, they are not considered to be the same since the rim appearance on both rims is uneven. Because it is well recognized among ophthalmologists that changes in the retinal rim are often the first indicators of glaucoma, it is only logical that a disc interpretation system should include the neuroretina rim as a unit of measurement.

Figure 1 represents different glaucoma. Located between the disc and the cup, the neuroretina rim acts as an external barrier to the outer margin of the optic nerve head, protecting it from external influences. Glaucoma is characterized by changes in the contour of the rim of the eyeball as a result of nerve damage in the eyeball itself. Therefore, the disc shape may be utilized in the early stages of diagnosis in order to reduce the misclassification bias produced by variances in disc size. Accurate segmentation of the OD and cup is necessary in order to provide a more specific localization of the neuroretina rim and, as a result, to allow for the development of innovative glaucoma evaluation methodologies. The majority of the time, damage in the glaucomatous eye was detected using OD measures, such as the OD and cup area, which have been previously discussed in this paper. When using shape-based approaches, the vast majority of them assume that the OD has been accurately divided and shaped. However, even a minor error in these segmentation-based methods might result in significant changes in the measurements and mistakes in the diagnosis of a patient's health, depending on the technique. The inability to objectively and quantitatively identify or predict the progression of glaucoma has persisted as a challenging obstacle to solve in recent years. It is crucial in the early detection and treatment of glaucoma that images generated via the use of imaging technologies be evaluated. Although such imaging methods have the potential to improve the accuracy of clinical assessment of retinal nerve fibers in the early stages of glaucoma, the accuracy of such assessments may be limited in the early stages of the disease due to a large number of overlaps and heterogeneity present in the retinal nerve fibers. It has been demonstrated that feature-based approaches outperform traditional methods in terms of diagnostic capabilities, though only a marginal improvement over standard methods has been demonstrated, and it is possible that they do not adequately capture local variation and unpredictable behavior in the retinal nerve fiber layer (RNFL). Consequently, an improved cost-effective glaucoma detection technique that relies on hybrid feature extraction from fundus photographs is proposed in this work. Through the extraction of histogram, texture, and fractal information from fundus photographs, the properties of fundus photographs are examined in the diagnosis of glaucoma. Below is a breakdown of the steps involved in developing the proposed hybrid features glaucoma diagnostic method.

The magnitude and phase characteristics of glaucoma are extracted in order to evaluate the early stages of the disease.

An examination of gray levels and the extraction of textural features were carried out in order to portray the physiological changes in fundus images [2] produced by the increase in cup size.

Fundus photographs are used to extract and evaluate the fractal properties of the region of interest in order to objectively investigate the morphological changes and complexity present in the region (ROI).

In order to increase the specificity and sensitivity of classification, we are examining and choosing differentiating aspects of glaucomatous pictures.

It is possible to automatically discriminate between normal and glaucoma eye photos using an adaptive neuro fuzzy inference system, which is based on the distribution of textural and fractal qualities (ANFIS). Following a specified clinical technique, the system may be used in conjunction with current ophthalmologic tests and clinical assessments. The fundus image analysis method proposed in this paper is an attempt to eliminate subjective variability by automating the analysis and minimizing the requirement for human participation from the operation as much as possible. The essay is split into three sections: the introduction, the background, and the approach. The introduction is broken into three sections: the results and outcomes of the experimental methods are presented in Section 4 of this paper. This is the section where you will find the conclusion.

## 2. Background

The effects of exposure to noise and other occurrences on medical images are well-known. The main aim of preprocessing an image is to enhance quality, reduce noise, resize the image for the required size, and so on. Prior to segmentation, one should first conduct a set of procedures aimed at addressing problems of noise, poor lighting, and retinal structures that affect the processing of the image. Because nonuniform illumination has a propensity to enhance contrast, nonuniform illumination may be corrected by using adaptive histogram equalization [3]. Segmentation is a procedure in which a signal is divided into meaningful components. Before the signal is segmented, research has been done to examine the ways to single out a channel. It is customary to use the red and green channels in order to segment OD and OC because they are very clearly represented in those channels. Morales et al. [4] used principal component analysis (PCA) to correlate pixel values across three color bands in order to help eliminate the influence of blood vessels on segmentation of OD, the results of which are shown in an improved image of the vascular tree. The Canny edge identification is then used to increase the distinction between vessels and nonvessels. Rodrigues et al. [5] utilized multiscale filtering based on Hessian using a genetic algorithm to get their optimum segmentation parameters for blood vessels. In Bharkad's research, he filtered the blood vessels and increased the optical depth area by using an equiripple low pass FIR filter [6].

Preprocessed image features are superior to raw image features. In kidneys, blood arteries are common, making it difficult to split them. Noise reduction and artery separation preprocessing can help with segmentation.

The Hough transform was shown to be efficient in separating OD in the red channel, as demonstrated by Hagiwara et al. [7]. Vessel displacement was computed using the chessboard metric, and several values were generated that allowed the diagnosis of normal and glaucoma fundus pictures. A new method was created that analyzes the flow of blood vessels in the optic nerve in order to identify and diagnose glaucoma. Using an intensity threshold, Rathore et al. [8] were able to compute clinical parameters for the first time by splitting the OD and OC. Bharkad et al. [6] utilized corner thresholding and point contour joining to segment the OD. According to Pardha Saradhi Mittapalli and Ahmadi et al. [9], a region-based active contour model takes into consideration restrictions on shape as well as other variables. Also, a novel segmentation method for optic cups is proposed based on structural and gray level properties. When separating OD levels, color and intensity data are included. This is done via the use of clustering, which uses the regional variations in the shade to assign a color to each separate section of the OC.

Shukla et al. [10] segregated optical density by minimizing the objective function for grouping pixels (OD). To segment the OC, thresholding is used using Otsu segmentation. Dey and Dey [11] utilized a randomized Hough transform in combination with a Canny edge detection technique to obtain optical contours in their research. To diagnose glaucoma, Gustian et al. [12] used a fully convolution network (FCN) and collected patient data and the contours of anatomical structure from case reports, and they were able to produce an image of the fundus. The authors of the work described in this paper used convolution neural networks to distinguish OC and OD pictures in their research, as Htay and Maung [13] reported. The filters provide data that is then sent to a softmax logistic classifier, which is a classifier that uses logistic regression.

Graph cut and convex hull procedures are used on the output of the classifier, which is segregated. In an effort to segment OD and OC pictures, Perdoma et al. built a deep neural network with 15 layers. The creation of a U-Net architecture was to help with the segmentation of OD and OC. This was done by Pandit et al. [14]. U-Net models have CNNs in them, and CNNs are the most vital part of a U-Net model. The latter of the two routes in this configuration grows, while the former shrinks. The contracting route is implemented using the architecture of CNN with resolution layers that work well. The expansion layer resolution is very low. The contracting path's image data is merged with the growing path's data. U-Net is able to identify patterns at a variety of scales.

Abbas [15] invented a hybrid strategy to identify the contours of OD and OC, which is also adaptively regularized and combines kernel-based fuzzy C-means (FCM) with the level set method to be able to differentiate between the two. Muthmainah et al. [16] invented a method for object classification utilizing superpixel classification, which classifies objects of interest (OD) and objects of concern (OC). Superpixel classification uses histogram features and statistical data to find the disc's boundary and is where OD segmentation starts.

Fine-tuning is possible by using a deformable model. To get the most accurate segmentation, the algorithm relies on local knowledge. In a study conducted by Caroline et al., active contour model (ACM) was combined with gradient vector flow (GVF) Yu et al. [17] to deal with the standard snake's flaws, including an inability to move into concave parts of the image during advancement and a limited range of capture. The external energy in snake equations is replaced by the internal energy in GVF with the use of edge gradients. The circular Hough transform is used to determine the snake's outline, the starting point of the analysis. After this, the snake is started with the OD boundary. In preparation for the snake's segmentation, GVF helps the snake regulate the OD boundary. A Hausdorff distance-based algorithm was used to locate the potential OD contours. Through the pyramidal decomposition method, it examines whether circular shapes may exist inside the different regions, just as a symbol might exist inside the OD. According to the study of Li et al. [18], an OD and OC segmentation contour-profiling model was developed to discover a category-based feature map optimization model that utilizes a region search to locate an optimal contour profile.

Muthmainah et al. [16] made progress in optical domain segmentation with the assistance of local binary patterns and density-based probability functions. To prevent segmentation mistakes, the red channel (which has a higher contrast) was segmented first, and all of the images were preprocessed with histogram equalization before being segmented. Pandit et al. [14] segmented the data for OD and OC by using a threshold technique. The author presents a multilevel thresholding approach for segmenting the image with fuzzy partitions of image histograms and entropy theory. In order to process the image, the RGB version of the picture is first converted into a grayscale version, and an image filtering technique is applied to reduce noise and enhance the results. The threshold for segmentation is determined using the Kapur test. Computing the CDR requires the use of the segmented OD and OC. The method for OD segmentation, as described by Tham et al. [19], involves the use of direction-based supervised learning between OD boundary coordinates, as well as a visual representation of OD, to show how it works. Kesarwani et al. [20] present a method for segmentation using a combination of CNN and dense-net methods. Convolutional blocks are densely connected together to form the pattern. The locally statistical ACM and a priori structure-based extraction is used to implement the model developed by Somogyi et al. [21] for OD and OC segmentation.

Hasan et al. present an article on end-to-end networks designed for segmentation and localization of OD and Fovea centers referred to as the DRNet. The method used was based on circular area searching. However, to estimate the OD radius, the method requires information about the camera's range of view. Cheng et al. presented their study, which includes a multiscale method for segmenting OD and OC. A creative CNN technique was used to create very dense feature maps, to get multiscale features. Features recovered by the pyramid filtering module via the pyramid filtering method. Bollwein and Westphal [22] proposed M-Net as a method for doing segmentation of OD and OC. The design of M-Net uses a multiscale input layer. To get a multilevel receptive field, an image pyramid is first created by downsampling images, which are then fed into the U-Net. The authors gave a multilabel loss to divide OD and OC based on the dice loss. Utama et al. [23] used a previously reported combination of RCNN to partition the OD and OC. Feature extraction begins with the VGG16 algorithm. Recovery of missing features and the subsequent split of the signal into the disc network and the cup network is performed by sending information via two divergent, parallel branches. In order to figure out where the OC should be placed, the system employs a disc attention module to parse the outcomes of the disc network and the cup network.

OC is hard to attain because of poor contrast, discontinuity of edges, and difficult-to-see OC and OD borders. A large number of techniques have similar effects on images with low contrast; they create under- and oversegmentation. Thresholding-based methods are more accurate than other methods to segment retinal images. Despite the potential to improve OD and OC segmentation, deformed models are adversely affected by bright exudates at the OD border and will likely fail to segment the fundus image because of their failure to adequately capture OD and OC segmentation. Based on the learning provided by CNN-based methods, the most accurate characteristics learned from the training data are then used to evaluate the test data. They require a large data set to train a CNN. Changing the demarcation of the OD and OC components has a huge effect on the CDR and NRR properties. A good way to fulfill this expectation is to invent a new kind of segmentation.

An artificial neural network for machine learning is a supervised classification system that may be distributed simultaneously and includes input and output components that are linked together through a weighted connection. The weights are modified to match the input samples in order to better forecast the class, according to results from research performed by David et al. Instance classifiers are also known as KNN algorithms. For a vote-based categorization, testing data is placed into several categories, which include but are not limited to location and other criteria.

Yu et al. [17] proposed a technique that relies on the Naïve Bayes theorem is used to classify exudates. Pixel-level descriptions are retrieved for each possible exudate region. Several new features were extracted from each pixel, and some of them were normalized with the average brightness of the optic disc in order to improve accuracy. Adaptive boosting is used to optimize Naïve Bayes classifiers for pixel classification.

A limited number of reports have surfaced that describe the use of deep learning algorithms, such as CNN, for object classification. Convolution, pooling, and dense connection are three steps of a network that use convolution. At the convolution and pooling layer, the feature extraction procedure reduces the sample dimensions.

In [24], how deep convolutional neural networks can be used to detect glaucoma in large screening campaigns using color fundus images is explored. The five architectures including standard CNN, VGG19, ResNet50, DENet, and GoogleNet performed well in terms of AUC, sensitivity, and specificity.

Tham et al. [19] presented a deep learning-based computer-aided diagnosis system for the detection of glaucomatous optic neuropathy (GON) on color fundus photographs.

It is possible that many distinct classifiers may make a range of errors on several samples. The model's constraints also include the requirement for large training data sets [25] as the number of layers in the CNN rises [26]. These problems may cause network settings to be improperly configured because of network degradation and issues such as missing information [27]. Using dynamic classifier selection techniques, an ensemble of classifiers may be generated to accommodate any misclassifications [28].

Based on the inference drawn from the literature, the research gaps identified are as follows:

- There is a lack of an effective preprocessing approach for accurate segmentation
- There is a lack of automated OD and OC segmentation techniques that overcome under- or oversegmentation due to the presence of exudates and low contrast between the boundaries

As part of the proposed work, fundus images will be used to identify anatomical structures along with pathological structures, and disease severity will be graded based on decision support tools to assist ophthalmologists.

## 3. Methodology of Proposed Work

Glaucoma is the second greatest cause of blindness and irreversible visual loss in the world, according to the World Health Organization. Glaucoma is sometimes referred to as “silent robbery of sight” by medical professionals since it destroys the optic nerve head and impairs peripheral vision as a result of the damage [19]. The early detection and categorization of glaucoma will enable patients to obtain proper treatment and assistance from their eye surgeons, which will improve their quality of life. A notable issue in health-care management exists because of the large number of prospective patients and the restricted number of ophthalmologists who are accessible to treat them. An early detection strategy for glaucoma is proposed in this proposed work to aid an ophthalmologist in the early diagnosis of the disease.

An image is processed by a deep convolutional neural network, which is typically used to detect low-, mid-, and high-level characteristics.

### 3.1. Retinal Image Data Set and Preprocessing

In order to verify the suggested structure, we used a private data set as well as three publicly available data sets.  Table 1 provides a high-level summary of the various data sources.

According to the picture containing the input, fundus is preprocessed using contrast limited histogram equalization (CLAHE) in order to improve image clarity. A minimum of 224 × 224 pixels is required for input dimensions in ResNet-50, GoogLeNet, and VGGNet-16 [29]. Following a contrast enhancement, the input picture is downsized from its original size of 224 × 224 pixels to 224 × 224 pixels. Deep learning requires a significant quantity of data to be effective, and this data must be collected in enormous quantities. Comprehensive training data are required for the development of an effective classifier, and they are also required for the improvement of the efficiency of a deep network. The process of data augmentation includes a range of methods such as rotational transformation, horizontal and vertical flipping, and other similar operations. It was necessary to employ an extra 6,955 photographs for the additional data gathering, which included flipping 1,391 images vertically, resulting in a total of three-turn transformations.

### 3.2. Feature Extraction from Pretrained CNN Architecture

Deep learning architectures VGGNet-16, ResNet-50, and GoogLeNet [30] are being studied, and each has its own set of advantages and disadvantages. Despite the fact that it is widely used for both general and medical image categorization, this architecture has been chosen. The next section contains in-depth discussions of each ConvNet design in detail.

#### 3.2.1. VGGNET-16

The VGGNet-16 architecture has 16 layers and is composed of two components. A 224 × 224 RGB picture is processed through a stack of convolution layers to produce a 224 × 224 RGB image. A picture is initially delivered to the top two layers, which are constructed of 64 channels of 3 × 3 filter sizes, before being transferred to the bottom two levels. A max pool layer of stride (2, 2) is followed by two layers of 3 × 3 filters and a convolution layer of 256 filters, all of which are applied after the max pool layer. This is followed by two sets of three convolution layers and a max pool layer, which are all repeated twice more. It is utilized in these convolution and max-pooling layers, rather than 7 × 7 and 11 × 11, a filter size of 3 × 3 is used instead. After each convolution layer, 1 pixel of padding is applied to prevent spatial characteristics in the picture from being seen.

The network architecture of VGGNet-16 can be seen in Figure 2. A stack of convolution layers is followed by three completely linked layers, which are then followed by another stack of convolution layers. The first layer is provided with a feature vector, and the first and second layers each have 4,096 channels, with the first layer having the most channels. The third layer, which is connected to the softmax layer, comprises 1,000 channels.

#### 3.2.2. ResNet-50

The residual network is a conventional neural network design that is used to tackle issues with vanishing gradients (vanishing gradient problems). Performance saturation and deterioration during backpropagation will arise as a consequence of repeated multiplication, which will result in a tiny gradient and performance saturation. ResNet was developed in order to avoid making connections. They enable the model to learn an identity function, which in turn allows for improved performance at the upper layer. Residual networks are a kind of deep convolution network that is composed of five stages, each of which has a convolution layer.

For the output block, feedforward neural networks with shortcut connections or a bottleneck design may be utilized to create the formula. In the first layer, an input consisting of a convolution of size 7 × 7 and 64 distinct kernels of size 2 are supplied. As well as these layers, a max-pooling layer with a stride size of 2 and a three-time convolution layer are included.  Table 2 has a more in-depth explanation of the ResNet-50 design.

The deep residual learning framework consists of function *f*(*a*) and *b* = *a* as identity mapping. The input to the block is added to the output block *F*(*a*) as follows:

(1) $$\begin{array}{c} F\left(a\right)=f\left(a\right)+a \end{array}$$

The cutoff influences achieve identity charting, and their productions are added to the outputs of the stacked layers, which is shown in Figure 3. These cutoffs help enhance the trainable parameters to improve the final performance of the network.

#### 3.2.3. GoogLeNet

The term GoogLeNet was introduced with a 22-layer network. Inception blocks use several smaller convolutional kernels to restrict the number of neurons and parameters. The GoogLeNet architecture is built up with 9 Inception modules (convolution kernels).  Figure 4 illustrates the underlying architecture for GoogLeNet.

The convolution procedure makes use of three different input filters, such as 1 × 1, 3 × 3, and 5 × 5. Before applying the convolution to the next inception module, the max-pooling operation is conducted on the convolution. The pooling layer was 5 × 5 with a stride of 3. The pooling layer was 5 × 5. Convolution with 128 filters for dimension reduction, as well as a rectified linear activation function, was used in the implementation. With a dropout layer that has a 70% dropout ratio, the suggested method achieves the desired results. Using a linear layer mixed with a softmax loss, it is possible to estimate the performance of the model.

### 3.3. Glaucoma Detection with Ensemble Model

The ensemble approach is a strong and fast method that develops numerous separate classification models and then combines them to improve accuracy. The proposed study uses three alternative ConvNet architectures: GoogLeNet, VGGNet-16, and ResNet-50, which are all variations of the GoogLeNet design. Several aspects of ConvNet, which is trained using data from the ImageNet data set, are shared by transfer learning as well. As a result, the ConvNet architecture is capable of learning generic characteristics without the need for further training. Deep features are recovered from the trained ConvNet architecture. To complete the process, ensemble characteristics are routed via a classifier layer in order to distinguish between normal and abnormal pictures, as shown in Figure 1.

## 4. Proposed Algorithm

This section presents a potential framework for glaucoma detection. Three benchmark data sets and one private data set were utilized to evaluate the proposed system's performance. Data sets are split into two categories: testing and training. The suggested ensemble model's flowchart is shown in Figure 5.

Following is a summary of the framework of the proposed algorithm:

**Step 1 .**

The algorithm starts with dividing the image samples into test and training samples

**Step 2 .**

Image preprocessing is performed initially on the fundus image in order to enhance some features, suppress falsification, and improve the image data

**Step 3 .**

After preprocessing, three different ConvNet architectures such as VGGNet-16, ResNet-50, and GoogLeNet were trained on the ImageNet data set

**Step 4 .**

The deep features are extracted from three ConvNet architectures

**Step 5 .**

Pretrained neural networks provide output that is combined into a prediction vector, and a decision is made based on majority voting

**Step 6 .**

Finally, digital fundus images are classified into normal and abnormal (glaucoma)

## 5. Results and Discussion

The proposed model is implemented with MATLAB 2020a software in an i7-7700K processor with 32 GB DDR4 RAM equipped with an NVIDIA GeForce GTX1060 3 GB Graphics Card. Performance measures for each deep learning architecture are evaluated using metrics such as accuracy, specificity, precision, sensitivity, and F1 score. The following equations provide the mathematical expressions of these parameters:

(2) $$\begin{array}{c} \text{Accuracy}=\frac{\text{TP}+\text{TN}}{\text{TP}+\text{TN}+\text{FP}+\text{FN}},\\ \text{Sensitivity}=\frac{\text{TP}}{\text{TP}+\text{FN}},\\ \text{Precision}=\frac{\text{TP}}{\text{TP}+\text{FP}},\\ \text{Specificity}=\frac{\text{TN}}{\text{TP}+\text{FP}},\\ F1\text{ score}=\frac{2{}^{*}\left(\text{Sensitivity}{}^{*}\text{Precision}\right)}{\left(\text{Sensitivity}+\text{Precision}\right)}, \end{array}$$

where the number of positive cases predicted correctly is TP, the number of negative cases predicted correctly is TN, the number of cases predicted incorrectly is FN when the case is negative, and the number of cases predicted incorrectly is FP when the case is positive.

The confusion matrix is shown in Figure 6, which depicts class 0 with a normal picture and class 1 with a glaucoma image. This architecture is tested against five distinct data sets: PSGIMSR (Polygonal Shaped Image Microstructure), HRF (Head and Neck Fracture), DRIONS-DB, DRISHTI-GS, and combined images. Four hundred and seventy-one pictures are determined to be normal, and 577 images are found to be aberrant in the PSGIMSR data set after a tenfold cross-validation is performed. There are 102 photos that have been misclassified.

Using the ResNet-50 architecture and VGGNet-16 and GoogLeNet architectures, the accuracy, precision, sensitivity, specificity, and F1 score were all improved. The results are provided in Table 3. Several data sets are used to compare the findings, including the PSGIMSR, the DRISHTI-GS, the DRIONS-DB, the HRF, and a merged data set.

It can be seen in Table 3 that the accuracy of the ResNet-50, VGGNet-16, and GoogLeNet architectures is 88.60%, 87.04%, and 86.86%, respectively, whereas the accuracy of the proposed architecture is 91.13% using the PSGIMSR data set, as can be seen in the results of the proposed architecture.

It is possible to attain the following sensitivity levels for the proposed method by using various data sets: 86.55%, 94.84%, 100%, 90.30%, and 81.26%. In order to assess the suggested framework, comparative studies are also carried out on a diverse variety of data sets.

The performance of ResNet-50, VGGNet-16, GoogLeNet, and proposed ensemble architecture was analyzed on five different data sets. From Figure 7, it is observed that the proposed ensemble architecture yields an accuracy of 91.13%, sensitivity of 86.37%, and specificity of 95.21% using the PSGIMSR data set. Maximum accuracy of 98.67%, sensitivity of 100%, and specificity of 97.4% is obtained using HRF (D3) data set. The combined data set (D5) yields an accuracy of 88.96%, sensitivity of 81.26%, and specificity of 95.53%.

Figure 8 shows the presentation of the future ensemble architecture in terms of F1 score using different data sets. From Figure 8, it can be stated that the proposed ensemble architecture outperforms ResNet-50, VGGNet-16, and GoogLeNet with the highest values of accuracy, sensitivity, specificity, precision, and F1 score.

## 6. Conclusion

In this proposed work, an ensemble model was designed for the detection of glaucoma in the early stage. In order to distinguish between normal and glaucomatous fundus pictures, the ensemble model proposes using a convolutional neural network to extract feature information from the images. The performance of the proposed method of ensemble architecture is compared with three ConvNet architectures such as ResNet-50, VGGNet-16, and GoogLeNet. The proposed approach is tested on various public and private data sets.

The performance of the proposed algorithm is better than the state-of-the-art technique. The proposed ensemble model yields an accuracy of 91.13%, sensitivity of 86.58%, and specificity of 95.21% using PSGIMSR data set; accuracy of 98.67%, sensitivity of 100%, and specificity of 97.40% using HRF data set. Experiments conducted on both public and private data sets show that the proposed model outperforms traditional computer-aided diagnosis algorithms and the convolutional neural network architecture. In this next proposed work, the investigation is carried out to design a fully convoluted network that can segment optic disc and optic cup with a large experimental data set.

## Figures and Tables

**Figure 1:** (a) Normal, (b) early glaucoma, (c) moderate glaucoma, and (d) severe glaucoma.

**Figure 2:** ConvNet architecture: VGGNet-16.

**Figure 3:** Learning methodology.

**Figure 4:** Block diagram of inception network.

**Figure 5:** Flowchart of the proposed ensemble model.

**Figure 6:** Confusion matrix of the binary classifier.

**Figure 7:** Comparison of accuracy of the proposed model.

**Figure 8:** Presentation contrast of the planned model: F1 score.

**Table 1:** Data set categorization.

Data set	Images		Resolution	Format
	Glaucoma	Normal		
**PSGIMSR**	650	500	720 × 576	JPEG
**DRISHTI-GS**	70	31	2,896 × 1,944	PNG
**DRIONS-DB**	60	50	600 × 400	JPEG
**HRF**	15	15	3,504 × 2,336	JPEG

**Table 2:** ConvNet configuration of ResNet-50

Layer name	ResNet-50	Output size
Conv 1	7 × 7, 64, stride 2	112 × 112
Conv 2	3 × 3 max pool, stride 2	56 × 56
	$\left[\begin{array}{cc} 1\times 1, & 64\\ 3\times 3, & 64\\ 1\times 1, & 256 \end{array}\right]$ × 3	
Conv 3	$\left[\begin{array}{cc} 1\times 1, & 128\\ 3\times 3, & 128\\ 1\times 1, & 512 \end{array}\right]$ × 4	28 × 28
Conv 4	$\left[\begin{array}{cc} 1\times 1, & 256\\ 3\times 3, & 256\\ 1\times 1, & 1024 \end{array}\right]$ × 6	14 × 14
Conv 5	$\left[\begin{array}{cc} 1\times 1, & 64\\ 3\times 3, & 64\\ 1\times 1, & 2048 \end{array}\right]$ × 3	7 × 7
Final	Average pool	1 × 1
	1,000, Fully connected	
	Softmax	

**Table 3:** Comparison of performance of proposed method for PSGIMSR with benchmark data sets.

Data set	Technique used	Accuracy	Precision	Sensitivity	Specificity	F1 score
**PSGIMSR (D1)**	GoogleNet	86.86	90.40	81.44	91.93	0.8568
	VGG	87.04	89.80	82.08	91.54	0.8576
	ResNet	88.60	91.60	83.72	93.03	0.8748
	**Proposed algorithm**	**91.11**	**94.18**	**86.55**	**95.20**	**0.9021**
**DRIONS-DB (D2)**	GoogleNet	90.90	90.80	89.37	92.22	0.9007
	VGG	91.63	90.40	91.12	92.05	0.9076
	ResNet	92.72	92.40	91.67	93.62	0.9203
	**Proposed algorithm**	**95.63**	**95.60**	**94.84**	**96.30**	**0.9521**
**HRF (D3)**	GoogleNet	95.33	94.67	95.94	94.73	0.9530
	VGG	96.00	97.33	94.80	97.26	0.9605
	ResNet	96.67	96.00	97.29	96.05	0.9664
	**Proposed algorithm**	**98.67**	**97.33**	**100**	**97.40**	**0.9864**
**Data set**	**Technique used**	**Accuracy**	**Precision**	**Sensitivity**	**Specificity**	**F1 score**
**DRISHTI-GS (D4)**	GoogleNet	92.07	89.03	85.71	95.05	0.8734
	VGG	91.08	87.09	84.37	94.20	0.8571
	ResNet	93.06	90.96	87.03	95.91	0.8895
	**Proposed algorithm**	**95.64**	**96.12**	**90.30**	**98.23**	**0.9312**
**Combined (D5)**	GoogleNet	83.40	87.50	75	90.69	0.8076
	VGG	83.73	86.87	75.81	90.38	0.8097
	ResNet	85.56	89.16	77.81	92.06	0.8310
	**Proposed algorithm**	**88.96**	**93.95**	**81.26**	**95.53**	**0.8714**

Bold represents the proposed algorithm values.

## Data Availability

The data that support the findings of this study are available on request from the corresponding author.
